The article "Circular RNA CNOT2 knockdown regulates twist family BHLH transcription factor via targeting microRNA 409-3p to prevent breast cancer invasion, migration and epithelial–mesenchymal transition" was retracted in 2024. Reasons: original data or images not available; unreliable results or conclusions; concerns about the data; concerns about the results or conclusions.

# Circular RNA CNOT2 knockdown regulates twist family BHLH transcription factor via targeting microRNA 409-3p to prevent breast cancer invasion, migration and epithelial–mesenchymal transition

**DOI:** 10.1080/21655979.2021.1974805

**Published:** 2021-10-26

**Authors:** QunXue Su, Hao Shen, Bei Gu, Ning Zhu

**Affiliations:** a Department of Pathology, Kunshan Second People’s Hospital, Kunshan City, China; b Department of Breast, Kunshan Second People’s Hospital, Kunshan City, JiangSu Province, 215300, China

**Keywords:** CircularRNA CNOT2, MicroRNA-409-3p, Twist Family BHLH Transcription Factor, Breast cancer, Epithelial–mesenchymal transition

## Abstract

Numerous studies have manifested that cicular RNA (circRNA) is closely associated with the development of breast cancer (BC), but the specific mechanism has not been fully clarified. The purpose of this study was to investigate the effect of circCNOT2 on BC invasion, migration and epithelial mesenchymal transition (EMT) and its potential molecular mechanism. The results assured that circCNOT2 and Twist Family BHLH Transcription Factor (TWIST1) were elevated in BC, while microrNA (miR)-409-3p was reduced. CircCNOT2 was positively correlated with TWIST1 and negatively correlated with miR-409-3p. Elevated circCNOT2 is associated with poor prognosis of BC. Knockdown circCNOT2 or augmented miR-409-3p could promote apoptosis but repress proliferation, invasion, migration and EMT of BC cells. In addition, overexpression of circCNOT2 or TWIST1 accelerated BC invasion, migration and EMT, which could be reversed by simultaneous transfection of miR-409-3p-mimic. Further dual luciferase reporting and RNA-pull down assay clarified that circCNOT2 acted as a competing endogenous RNA of miR-409-3p to mediate TWIST1 expression. In conclusion, the results of this study suggest that circCNOT2 affects the biological behavior of BC via regulating the miR-409-3p/TWIST1 axis, and may be applied as a potential therapeutic target for BC later.

## 1. Introduction

Breast cancer (BC), the most universal cancer in females, has become a serious public health problem worldwide [1]. Studies have shown that its mortality accounts for 14% of the total among female cancer [2]. In recent years, BC incidence has an year-by-year increase. Since 2008, BC-related mortality has elevated by nearly 18% [3]. Although measures including drugs, radiation therapy and surgery can alleviate BC development, its survival rate is still low with large side effects [4]. Therefore, it is necessary to further probe into the molecular mechanism of BC pathogenesis to seek key targets for effective treatment.

CircularRNA (circRNA) is an endogenous RNA that has been re-recognized in recent years. As high-throughput sequencing and bioinformatics develop, increasing circRNAs have been identified in eukaryotic transcriptome. Via combining with miRNA, it plays a key role in regulating transcription and post-transcriptional gene expression [5]. A great many studies have supported that circRNA affects various diseases, like cardiovascular diseases, cancer and neurological diseases [6,7]. Recently, based on ever-growing studies, circRNA is crucial in treating and diagnosing BC [8,9]. CircCNOT2, a recently identified circRNA, is highly expressed in BC. Its knockdown is available to signally repress BCMCF-7 and BT474 cell viability [10]. But migration, invasion and EMT are vital factors for evaluating cancer metastasis [11]. Whether Circ _CNOT2 takes part in regulating BC migration, invasion and EMT and its specific mechanism has not been ascertained.

The article "Circular RNA CNOT2 knockdown regulates twist family BHLH transcription factor via targeting microRNA 409-3p to prevent breast cancer invasion, migration and epithelial–mesenchymal transition" was retracted in 2024. Reasons: original data or images not available; unreliable results or conclusions; concerns about the data; concerns about the results or conclusions.

Thus, this study was implemented to probe into the changes in BC cell invasion, migration and EMT after silencing circCNOT2 via constructing siRNA that targets circCNOT2. Additionally, DLR and RNA-pull down experiments supported that downstream miRNA and target genes received impacts from circCNOT2 amid BC progression, thus providing a further theoretical basis for diagnosing and treating BC.

## 2 Methods and materials

### 2.1. Tissue sample collection

Total 44-pair BC tissue and adjacent normal tissue samples were gained from patients who received treatment from 2012–2014 in Kunshan Second People’s Hospital. Patients’ clinicopathological characteristics were collected for further evaluation. All patients in this study voluntarily signed written informed consent. Additionally, the study has got approval from the Human Research Ethics Committee of Kunshan Second People’s Hospital.

### 2.2. Cell culture

Human normal breast epithelial cell line (MCF-10A) and two human BC cell lines (MCF-7, SKBR-3) were bought from the Chinese Academy of Sciences (Shanghai, China). All cell lines were given culture in RPMI1640 medium (Gibco, U.S.) with 10% fetal bovine serum (FBS, Invitrogen), 100 IU/mL penicillin and 100 mg/mL streptomycin (Abcam, UK) at 37°C in a humid surrounding containing 5% CO_2_.

### 2.3. Cell transfection

For circCNOT2 knockdown, small interfering RNA (siRNA) targeting circCNOT2 (si-CNOT2) was synthesized with si-negative control (NC) (Genepharma, Shanghai, China) as a NC. Additionally, overexpressed plasmids targeting circCNOT2 and TWIST1 (oe-CNOT2/TWIST1) and elevated plasmid NCs (oe-NC) were bought from Genepharma. Aiming to enrich miR-409-3p, miR-409-3p-mimic and mimic-NC were bought from Ribobio (Guangzhou). Cell transfection was done in BC cells via Lipofectamine 3000 (Invitrogen, U.S.) [12].

The article "Circular RNA CNOT2 knockdown regulates twist family BHLH transcription factor via targeting microRNA 409-3p to prevent breast cancer invasion, migration and epithelial–mesenchymal transition" was retracted in 2024. Reasons: original data or images not available; unreliable results or conclusions; concerns about the data; concerns about the results or conclusions.

### 2.4. 3-(4,5-dimethyl-2-thiazoly)-2,5-diphenyltetrazolium bromide (MTT) determination

In reference to manufacturer’s request, transfected MCF-7 cells (2000 cells/well) proliferation was tested at different times (24, 48 and 72 h) using MTT cell proliferation assay kit (Sangon Biotech, China). Absorbance measurement was done at 490 nm under microplate reader (Thermo Fisher Scientific, Massachusetts, USA).

### 2.5. Flow cytometry

Via Annexin V Apoptosis Detection Kit (Sangon Biotech) MCF-7 cell apoptosis was studied, that is, these cells were treated with resuspension in 195 μL of binding buffer (4 × 10^5^ cells), later exposed to AV-FITC for 15 minutes, and treated with 10 μL of propidium iodide. At last, apoptotic cells were identified via flow cytometry (BD Bioscience, U.S.).

### 2.6. Transwell migration assay

The cell migration was detected as set forth [13]. Transwell chamber (Corning, U.S.) was applied in this assay. BC cells were subjected to seeding into upper chambers with serum-free Dulbecco’s Modified Eagle Medium (DMEM). Meanwhile, DMEM containing 20% FBS was added to lower chambers. After 24 hours, cell removal in upper chambers was done with cotton swabs, while cells in surface of lower chambers were subjected to fixation with 4% paraformaldehyde (PFA) to stain with 0.1% crystal violet for 15 minutes. After wash twice with PBS, the number of cells in five selected areas by random under microscopes was counted (Olympus, Japan).

### 2.7. Transwell invasion assay

Transwell upper chambers (Corning) coated with diluted Martrigel (BD Bioscience) and serum-free DMEM, were employed to seed MCF-7 cells, and later were treated with incubation in DMEM wells containing 10% FBS. After 24-hour incubation at 37°C, cells in inner chambers and remaining Matrigel were subjected to removal with cotton swabs, whereas cells on surface of lower chamber outsides were treated with fixation with 4% PFA to stain with 0.1% crystal violet for 15 minutes. After wash twice with PBS, the number of cells in five selected areas by random was counted under microscopes.

### 2.8. Reverse transcription quantitative polymerase chain reaction (RT-qPCR)

TriQuick Reagent (Solarbio, China) was applied to extract total RNA from BC tissue samples and cells. Via random primers (TaKaRa, China) for reverse transcription of circCNOT2 and TWIST1, and miRNA 1st cDNA synthesis kit (Vazyme, Nanjing, China) for that of miR-409-3p, qPCR was done on ABI 7500 RealTime PCR system (Applied Biosystems, U.S.) via SYBR Premix Ex Taq II (TaKaRa). Relative circRNA, mRNA and miRNA expression levels were subjected to calculattion in reference to 2^−ΔΔCt^. U6 was applied as the internal reference for miRNA and glyceraldehyde-3-phosphate dehydrogenase (GAPDH) for mRNA.each experiment was repeated three times, primer sequences detailed in Table 1.

The article "Circular RNA CNOT2 knockdown regulates twist family BHLH transcription factor via targeting microRNA 409-3p to prevent breast cancer invasion, migration and epithelial–mesenchymal transition" was retracted in 2024. Reasons: original data or images not available; unreliable results or conclusions; concerns about the data; concerns about the results or conclusions.

**Table 1.** RT-qPCR primer sequences

	Primer sequences (5′ – 3′)
GAPDH	Forward: 5ʹ-ATGGGGAAGGTGAAGGTCG-3’
	Reverse: 5ʹ-TTACTCCTTGGAGGCCATGTG-3’
U6	Forward: 5ʹ-CTCGCTTCGGCAGCACATATACT-3’
	Reverse: 5ʹ-ACGCTTCACGAATTTGCGTGTC-3’
CircCNOT2	Forward: 5ʹ-TCCACATCGGTCAGAAAAAGAT-3’
	Reverse: 5ʹ- GAGGCAATCAAATAGAACTGTCACT −3’
miR-409-3p	Forward: 5ʹ-GAATGTTGCTCGGTGA-3’
	Reverse: 5ʹ-GTGCAGGGTCCGAGGT-3’
TWIST1	Forward: 5ʹ- GCCAGGTACATCGACTTCCTCT −3’
	Reverse: 5ʹ-TCCATCCTCCAGACCGAGAAGG-3’

### 2.9. Western blot

In short, Radio-Immunoprecipitation assay buffer (Solarbio) was employed to do total protein extraction from cells or tissues. Concentration of protein sample was evaluated via Pierce bicinchoninic acid protein detection kit (Termo Scientifc, U.S.). In equal amount, 30 μg protein sample separation was done via sulfate polyacrylamide gel electrophoresis to transfer to Polyvinylidene fluoride films that were later subjected to block in skim milk at room temperature for 2 h and incubated with primary antibodies: GAPDH (sc-32,233, 1:1000, Santa Cruz Biotechnology), E-cadherin (20,874-1-AP, 1:1000, Proteintech), N-cadherin (13,116, 1:1000, Cell Signaling Technology), Vimentin (5741, 1:1000: Cell Signaling Technology), Snail (ab53519, 1:1000, Abcam), TWIST1 (sc-81,417, 1:1000, Santa Cruz Biotechnology) overnight at 4°C. After the films were treated with incubation with goat anti-rabbit Immunoglobulin G-horseradish peroxidase secondary antibody (Abcam) at 37°C for 2 hours, protein signal visualization was done via eyoECL plus kit (Beyotime, China).

### 2.10. Double luciferase reporter (DLR) experiment

Through online database starbase (http://starbase.sysu.edu.cn/) for bioinformatics analysis, predicting the interaction was between miR-409-3p and circCNOT2 or TWIST1 to analyze their binding sites; Based on predicted sequence-WT of binding sites, sequence-MUT of circCNOT2 and TWIST1 mutating at binding sites were designed. Later, the two kinds of sequences were treated with amplification and clone into PGL4 reporter plasmids (Promega, U.S.), that is, circCNOT2-WT, circCNOT2-MUT, TWIST1-WT and TWIST1-MUT. Quickly, separated fusion plasmids and miR-409-3p-mimic or mimic-NC were treated with co-transfection into MCF-7 cells. After 48 hours, luciferase activity detection was done on dual luciferase assay system (Promega).

### 2.11. RNA-pull down

MiR-409-3p and mimic-NC labeled with biotin from Ribobio were named Biotin-miR-409-3p and Biotin-mimic-NC, respectively, and were treated with transfection into MCF-7 cells and 48-hour incubation, after which the cells were placed in lysis buffer. Pierce Magnetic RNA Protein Pulldown Kit (Thermo Fisher Scientific) was later employed for determination. RNA abundance was checked via RT-qPCR analysis.

The article "Circular RNA CNOT2 knockdown regulates twist family BHLH transcription factor via targeting microRNA 409-3p to prevent breast cancer invasion, migration and epithelial–mesenchymal transition" was retracted in 2024. Reasons: original data or images not available; unreliable results or conclusions; concerns about the data; concerns about the results or conclusions.

### 2.12. Statistics

The data were expressed as mean ± standard deviation. The Student’s t test was applied to determine the statistical significance of the difference between the two groups, while the χ2 test to assess the correlation between circCNOT2 levels and clinical features. Prism Software 8.0 (GraphPad Software, USA) was employed to analyze and display the data. *P < 0.05 was considered to be a statistically significant difference.。 At least three biological replicates were performed for all the results of this study, and three technical replicates for each biological sample.

## 3 Results

### 3.1. CircCNOT2 is up-regulated in BC

To explore the biological function of circCNOT2 in BC, CNOT2 expression was checked in BC. Vs. adjacent normal tissues, CNOT2 was signally up-regulated in BC tissues, which is consistent with previous findings (Figure 1a). For further confirmation, CNOT2 expression was analyzed in MCF-7 and SKBR-3 and MCF-10A. In the latter, CNOT2 level was signally higher (Figure 1b). In reference to the median of CNOT2 expression (3.82times, fold change to normal tissue), the patients were allocated into high expression group and low expression group, and correlation analysis of clinicopathological characteristics was done, finding that CNOT2 was highly correlated with TNM staging and tumor size (Table 2). Additionally, Kaplan–Meier survival curve of BC patients revealed that BC patients’ survival prognosis with high CNOT2 expression was visually worse than those with low (Figure 1c). These findings indicate that circCNOT2 expression elevates in BC, which is related to poor survival prognosis.

**Table 2.** Correlation analysis of circCNOT2 and clinicopathological characteristics of BC patients

Characteristics	Groups	Cases	MiR-409-3p expression		P
			High expression group (n = 22)	Low expression group (n = 22)	
Age	< 60	17	10 (45%)	7 (31%)	0.3530
	60 or more	27	12 (55%)	15 (69%)	
Gener	Male	21	9 (40%)	12 (55%)	0.3652
	Female	23	13 (60%)	10 (45%)	
Tumor size (cm)	< 5 cm	19	3 (13%)	16 (72%)	<0.0001
	5 cm or more	25	19 (87%)	6 (28%)	
Histological grade	Moderate	30	14 (63%)	16 (72%)	0.5174
	Low	14	8 (37%)	6 (28%)	
TNM staging	I + II	13	3 (13%)	10 (45%)	0.0207
	III + IV	31	19 (87)	12 (55%)

**Figure 1.** **Up-regulated circCNOT2 in BC is linked with poor prognosis**. A: RT-qPCR to detect circCNOT2 expression in BC tissue samples and adjacent normal tissues; B: RT-qPCR to detect circCNOT2 expression in MCF-10A and MCF-7 and SKBR-3; C: Prognostic chart of patients with high-expression circCNOT2 and low-expression circCNOT2. Values presentation was detailed in mean ± SD (n = 3). Via one-way ANOVA to calculate the significance of each group, the variance correction was done via Tukey’s test. *P < 0.05

The article "Circular RNA CNOT2 knockdown regulates twist family BHLH transcription factor via targeting microRNA 409-3p to prevent breast cancer invasion, migration and epithelial–mesenchymal transition" was retracted in 2024. Reasons: original data or images not available; unreliable results or conclusions; concerns about the data; concerns about the results or conclusions.

### 3.2. Knocking down circCNOT2 effectively prevents BC invasion, migration and EMT

Aiming to probe into how CNOT2 biologically functions in BC, MCF-7 cells was selected with the highest expression level for subsequent experiments. After transfecting si-CNOT2, CNOT2 level in MCF-7 was obviously reduced (Figure 2a). Later, the impacts of knocking down CNOT2 was examined on proliferation, apoptosis, migration, invasion and EMT in MCF-7 cells, finding that this knockdown effectively inhibited proliferation (Figure 2b). Flow cytometry revealed that such knockdown observably promoted apoptosis (Figure 2c). Additionally, Transwell assay implied that this knockdown reduced invasion and migration ability (Figure 2d). Based on western blot findings, knocking down CNOT2 also increased E-cadherin expression but inhibited N-cadherin, Vimentin and snail expressions (Figure 2e). These findings indicate that circCNOT2 knockdown effectively prevents BC from deterioration.

**Figure 2.** **CircCNOT2 knockdown effectively prevents BC invasion, migration and EMT**. A: RT-qPCR to detect the impact of circCNOT2 knockdown on MCF-7 cells; B: MTT to detect the impact of circCNOT2 knockdown on MCF-7 cell proliferation; C: Flow cytometry to detect the impact of circCNOT2 knockdown on MCF-7 apoptosis; D: Transwell to detect the effect of knocking down circCNOT2 on the of MCF-7 cell invasion and migration; E: Western blot to detect the effect of knocking down circCNOT2 on E-cadherin, N-cadherin, Vimentin and snail protein expressions in MCF-7 cells. Values presentation was detailed in mean ± SD (n = 3). Via one-way ANOVA to calculate the significance of each group, the variance correction was done via Tukey’s test. *P < 0.05

### 3.3. CircCNOT2 competitively bind to miR-409-3p

CircRNA usually functions in cancer as a miRNA sponge [14]. Next, the downstream miRNA binding to circCNOT2 was exploited. A miRNA was noticed namely miR-409-3p, has proved to be under-expressed in BC and low-level miR-409-3p links with the poor prognosis of BC [15]. First check of its expression level was in BC. MiR-409-3p expression was signally reduced in BC patients (Figure 3a). Additionally, the same findings existed in cell experiments. MiR-409-3p level in two BC cell lines was visually lower than that of MCF-10A cells (Figure 3b). Later, whether miR-409-3p is regulated by circCNOT2 was checked in BC. After knocking down or overexpressing circCNOT2, miR-409-3p level in MCF-7 cells was signally elevated or lowered, respectively (Figure 3c). Consequently, it was speculated that miR-409-3p maybe target circCNOT2. Aiming to prove this conjecture, it was predicted that circCNOT2 and miR-409-3p have specific binding sites through bioinformatics website http://starbase.sysu.edu.cn/ (Figure 3d). DLR experiment showed that CNOT2-WT significantly reduced dual-luciferase activity of miR-409-3p-mimic group, wherea CNOT2-MUT had no obvious impact on it (Figure 3e). Additionally, RNA-pull down experiment revealed that biotinylated miR-409-3p successfully captured circCNOT2, indicating that miR-409-3p and circCNOT2 interacted with each other (figure 3f). What’s more, the correlation analysis on miR-409-3p expression and circCNOT2 revealed that they had a negative correlation (Figure 3g). These findings indicate that circCNOT2 competitively binds to miR-409-3p in BC.

The article "Circular RNA CNOT2 knockdown regulates twist family BHLH transcription factor via targeting microRNA 409-3p to prevent breast cancer invasion, migration and epithelial–mesenchymal transition" was retracted in 2024. Reasons: original data or images not available; unreliable results or conclusions; concerns about the data; concerns about the results or conclusions.

**Figure 3.** **CircCNOT2 competitively binds to miR-409-3p**. A: RT-qPCR to detect miR-409-3p expression in BC and adjacent normal tissues; B: RT-qPCR to detect miR-409-3p expression in MCF-10A, MCF-7 and SKBR-3; C: RT-qPCR to detect the influence of knocking down or overexpressing circCNOT2 on miR-409-3p expression; D: Via http://starbase.sysu.edu.cn/ to predict binding sites of circCNOT2 and miR- 409-3p; E-F: DLR and RNA-pull down experiments to detect the targeting relationship between circCNOT2 and miR-409-3p, respectively; G: Correlation analysis on circCNOT2 and miR-409-3p expressions in patients’ tissues. Values presentation was detailed in mean ± SD (n = 3). Via one-way ANOVA to calculate the significance of each group, the variance correction was done via Tukey’s test. *P < 0.05

### 3.4. Overexpressing miR-409-3p inhibits BC invasion, migration and EMT

Next, it was probed into how miR-409-3p biologically acts in BC. By transfecting miR-409-3p-mimic, up-regulated miR-409-3p was in MCF-7 cells (Figure 4a) to checked its effects on MCF-7 cell proliferation, apoptosis, invasion, migration, and EMT. Overexpressing miR-409-3p signally inhibited proliferation and elevated apoptosis rate (Figure 4b and 4c). Transwell implied that overexpressing miR-409-3p effectively reduced invasion and migration (Figure 4d). Additionally, RT-qPCR and western blot findings supported that overexpressing miR-409-3p elevated E-cadherin expressions in MCF-7 cells but inhibited N-cadherin, Vimentin and snail expression (Figure 4e). These findings indicate that miR-409-3p as a tumor suppressor gene in BC effectively inhibits BC cell invasion, migration and EMT.

**Figure 4.** **Overexpressed miR-409-3p inhibits BC invasion, migration and EMT**. A: RT-qPCR to detect the impact of overexpressing miR-409-3p on MCF-7 cell; B: MTT method to detect the influence of overexpressing miR-409-3p on MCF-7 cell proliferation; C: Flow cytometry to detect the impact of overexpressing miR-409-3p on MCF-7 cell apoptosis; D: Transwell to detect the effect of overexpression of miR-409-3p on MCF-7 cell invasion and migration; E: Western blot to detect the impact of overexpressing miR-409-3p on E-cadherin, N-cadherin, Vimentin and snail protein expression in MCF-7 cells. Values presentation was detailed in mean ± SD (n = 3). Via one-way ANOVA to calculate the significance of each group, the variance correction was done via Tukey’s test. *P < 0.05

The article "Circular RNA CNOT2 knockdown regulates twist family BHLH transcription factor via targeting microRNA 409-3p to prevent breast cancer invasion, migration and epithelial–mesenchymal transition" was retracted in 2024. Reasons: original data or images not available; unreliable results or conclusions; concerns about the data; concerns about the results or conclusions.

### 3.5. TWIST1 is a target gene of miR-409-3p

TWIST1 has proved to be up-regulated in BC, which links with BC EMT [16]. So it waschecked whether it is a target gene of miR-409-3p. In BC patients’ cells, TWIST1 expression was visually elevated, which is consistent with previous findings (Figure 5a and 5b) [17]. Additionally, it was found that in MCF-7 cells, up-regulated miR-409-3p effectively inhibited TWIST1 expression (Figure 5c). Consequently, it was speculated that TWIST1 may be a potential target gene of miR-409-3p. Aiming to verify this conjecture, a prediction through bioinformatics website http://starbase.sysu.edu.cn/ was that TWIST1 and miR-409-3p had specific binding sites (Figure 5d). To further support our conjecture, DLR and RNA-pull down experiments were done, finding that TWIST1-WT effectively repressed the dual luciferase activity of miR-409-3p-mimic group. Additionally, biotinylated miR-409-3p-mimic successfully captured TWIST1 (Figure 5e and 5f). In correlation analysis, patient’s TWIST1 and miR-409-3p levels were negatively correlated (Figure 5g). These data indicate that TWIST1 may be a potential target gene of miR-409-3p.

**Figure 5.** **TWIST1 is a target gene of miR-409-3p**. A: RT-qPCR to detect TWIST1 expression in BC tissue samples and adjacent normal tissues; B: RT-qPCR and western blot to detect TWIST1 expression in MCF-10A, MCF-7 and SKBR-3 C: RT-qPCR and western blot to detect how up-regulated miR-409-3p impacted TWIST1; D: Via http://starbase.sysu.edu.cn/ to predict the binding sites of TWIST1 and miR-409-3p; E-F: DLR and RNA-pull down experiments to detect the targeting relationship between TWIST1 and miR-409-3p, respectively; G: Correlation analysis on TWIST1 and miR-409-3p expressions. Values presentation was detailed in mean ± SD (n = 3). Via one-way ANOVA to calculate the significance of each group, the variance correction was done via Tukey’s test. *P < 0.05

The article "Circular RNA CNOT2 knockdown regulates twist family BHLH transcription factor via targeting microRNA 409-3p to prevent breast cancer invasion, migration and epithelial–mesenchymal transition" was retracted in 2024. Reasons: original data or images not available; unreliable results or conclusions; concerns about the data; concerns about the results or conclusions.

### 3.6. Up-regulated TWIST1 promotes BC cell invasion, migration and EMT

Later, overexpressed TWIST1 was in MCF-7 cells (Figure 6a) to examine its impact on BC cell proliferation, apoptosis, invasion and migration and EMT. After up-regulating TWIST1, MCF-7 cell proliferation was signally elevated but its apoptosis rate was visually reduced (Figure 6b and 6c). Additionally, Transwell findings revealed that up-regulated TWIST1 signally promoted MCF-7 cell invasion and migration (Figure 6d). Based on RT-qPCR and western blot, up-regulated TWIST1 reduced E-cadherin expression in MCF-7 cells but elevated N-cadherin, Vimentin and snail expression (Figure 6e). This indicates that up-regulated TWIST1 promotes BC cell proliferation, invasion, migration and EMT, thus inhibiting apoptosis.

**Figure 6.** **Up-regulated TWIST1 promotes BC cell invasion, migration and EMT**. A: RT-qPCR and western blot to detect how up-regulated TWIST1 influenced MCF-7 cell; B: MTT method to detect how up-regulated TWIST1 impacted MCF-7 cell proliferation; C: Flow cytometry to detect the impact of up-regulated TWIST1 on MCF-7 cell apoptosis; D: Transwell to detect the influence of up-regulated TWIST1 on MCF-7 cell invasion and migration; E: Western blot to detect the impact of up-regulated TWIST1 on E-cadherin, N-cadherin, Vimentin and snail protein expression in MCF-7 cells. Values presentation was detailed in mean ± SD (n = 3). Via one-way ANOVA to calculate the significance of each group, the variance correction was done via Tukey’s test. *P < 0.05

### 3.7. MiR-409-3p/TWIST1 axis is involved in circCNOT2’s regulating on BC

Finally, it was probed into whether miR-409-3p/TWIST1 takes part in the process of circCNOT2 regulating on BC. In BC patients, TWIST1 level and circCNOT2 expression were positively correlated (Figure 7a). Later, miR-409-3p was overexpressed while overexpressing circCNOT2, finding that the latter signally increased circCNOT2 and TWIST1 expression, whereas TWIST1 level was signally reversed after miR-409-3p-mimic treated with simutaneous transfection (Figure 7b). Subsequently, it was examined what impacts the co-transfection imposed on BC biological functions. Overexpressed circCNOT2 visually elevated the of MCF-7 cell proliferation but inhibited its apoptosis, whereas promoted its invasion and migration capabilities, reducing E-cadherin expression and promoting N-cadherin, Vimentin and snail expression (Figure 7c-f). Simultaneous transfection of miR-409-3p-mimic reversed the impact posed by overexpressing circCNOT2 on MCF-7 cell proliferation, apoptosis, invasion, migration and EMT. This indicates that circCNOT2 affects BC proliferation, apoptosis, invasion and migration and EMT via regulating miR-409-3p/TWIST1 axis.

The article "Circular RNA CNOT2 knockdown regulates twist family BHLH transcription factor via targeting microRNA 409-3p to prevent breast cancer invasion, migration and epithelial–mesenchymal transition" was retracted in 2024. Reasons: original data or images not available; unreliable results or conclusions; concerns about the data; concerns about the results or conclusions.

**Figure 7.** **MiR-409-3p/TWIST1 axis is involved in the process of circCNOT2 regulating on BC**. A: Correlation analysis on TWIST1 and circCNOT2 expressions in patients’ tissues; B: RT-qPCR and western blot to detect how co-transfection impacted circCNOT2 and TWIST1 expressions; C: MTT to detect the influence of co-transfection on MCF-7 cell proliferation; D: Flow cytometry to detect how co-transfection affected MCF-7 cell apoptosis; E: Transwell to detect the impact of co-transfection on MCF-7 cell invasion and migration; F: Western blot to detect how co-transfection impacted E-cadherin, N-cadherin, Vimentin and snail protein expression in MCF-7 cells. Values presentation was detailed in mean ± SD (n = 3). Via one-way ANOVA to calculate the significance of each group, the variance correction was done via Tukey’s test. *P < 0.05

## 4. Discussion

BC, among the most common cancers in women, is very aggressive with high mortality [18]. A great many studies have revealed that circRNA is involved in regulating post-transcriptional expression in human body, playing an essential role in cancer occurrence and development [19]. In this study, it was found that circCNOT2 affects BC cell proliferation, migration, invasion and EMT via regulating miR-409-3p/TWIST1 axis.

Based on previous studies, with high stability in tissues and blood, circRNA usually acts as a potential biomarker for cancer prognosis and diagnosis [20]. In this study, it was demonstrated that circCNOT2 expression was up-regulated in BC tissues and was extremely correlated with clinicopathologic features and poor postoperative prognosis of BC. However, its expression in the serum of patients remains unclear. It is necessary to detect circCNOT2 expression in the serum of patients in subsequent experiments, which is crucial to determine whether circCNOT2 can be applied as an early biomarker for BC diagnosis. Recent studies have reported that various circRNAs are abnormally expressed in BC and participate in BC development. For example, Liu C *et al*. found 520 circRNAs that are abnormally expressed in BC, among which hsa_circ_0043278 expression is relative to patient’s lymph node metastasis and histological type. This study manifested that circCNOT2 is largely correlated with patient’s TNM staging and tumor size. Additionally, high-level circCNOT2 has a worse prognosis, which is consistent with previous findings. Smid M *et al*. also clarified that inhibiting CNOT2 is available to attenuate BC cell proliferation. Wang F *et al*. reported that high-level circNOL10 inhibits BC cell proliferation, migration and invasion *in vitro* [21]. This supports that high- or low-level circRNA can affect BC development. In this study, it was observed that silencing circCNOT2 inhibited BC proliferation via regulating the miR-409-3p/TWIST1 axis. Additionally, it was also noticed that BC cell migration, invasion and EMT process are also under regulation by circCNOT2. This suggests that circCNOT2 is a key oncogenic element in BC. It is worth noting that the biological function and molecular mechanism of circCNOT2 were only explored in vitro experiments in this study, and the effect of knockdown circCNOT2 on BC tumors in vivo is still unclear, which needs to be explored in subsequent studies. In addition, only MCF-7 cells were applied in this study, and the role of circCNOT2 in other BC cell lines may be different. This is a limitation of this study.

The article "Circular RNA CNOT2 knockdown regulates twist family BHLH transcription factor via targeting microRNA 409-3p to prevent breast cancer invasion, migration and epithelial–mesenchymal transition" was retracted in 2024. Reasons: original data or images not available; unreliable results or conclusions; concerns about the data; concerns about the results or conclusions.

TWIST1 is a basic helix-loop-helix transcription factor encoded by the TWIST1 gene. It has proved that this factor is directly related to the pathogenesis of various diseases, like neurocognitive defects [22], intervertebral discs degeneration [23], osteoarthritis [24] and cancer [25,26]. Importantly, TWIST1 is usually seemed as a transcription factor of cancer EMT, playing an essential role in cancer metastasis [27]. Previous reports have revealed that the interaction between TWIST1 and various miRNAs take part in regulating cancer, like miR-16, miR-26b-5p, miR-1271, miR-539, miR-214, miR-200b/c, miR-335, miR-10b and miR-381, while TP73-AS1, LINC01638, ATB, NONHSAT101069, CASC15, H19, PVT1, LINC00339, LINC01385, TANAR, SNHG5, DANCR, CHRF and TUG1 are positively regulating TWIST1 and affects long non-coding RNA in carcinoma development [28]. This study testified that overexpressing TWIST1 promotes BC cell proliferation, migration, invasion and EMT, which is consistent with previous reports. Additionally, a new circRNA/miRNA axis (circCNOT2/miR-409-3p) was found to target TWIST1 expression in BC. This will provide new insights into TWIST1’s involvement in cancer pathogenesis.

## 5. Conclusion

To conclude, it was found that circCNOT2 and TWIST1 are highly expressed in BC, while miR-409-3p is under-expressed. BC patients with high-level circCNOT2 have worse prognosis. It was demonstrated for the first time that silencing circCNOT2 inhibits the of BC cell growth, migration, invasion and EMT via regulating the miR-409-3p/TWIST1 axis, thus providing a better understanding of BC pathogenesis and a possible target for treating BC.
